The article "Analysis of Improving Effect of Running APP on College Students' Physique by Using Student Data Mining Technology" was retracted in 2023. Reasons: suspected computer-generated content; unreliable results or conclusions; lack of ethics approval or compliance; missing or withdrawn patient consent.

# Analysis of Improving Effect of Running APP on College Students' Physique by Using Student Data Mining Technology

**DOI:** 10.1155/2022/4807953

**Published:** 2022-07-21

**Authors:** Ni Zhuo

**Affiliations:** Guangxi Electromechanical Vocational and Technical College, Nanning 530007, China

## Abstract

With the continuous development of sports software, college students, as the most advanced social new ideological group, running APP gradually enter the study and life of college students. Based on students' DM (data mining), this paper analyzes the influence of running apps on the improvement of college students' physique, chooses DT (decision tree) algorithm to construct the structure according to the characteristics of the data used, obtains students' DM model, and prunes it by using substitution error rate and PEP (pessimistic error pruning). The results show that the results of intra-group comparison among boys show that the scores of 1000 m in the intervention group have no obvious change compared with those before the intervention, and the difference is not statistically significant (*P*=0.516). The 800 m scores of girls in the intervention group were better than those in the control group, and the difference was statistically significant (*P*=0.03). The results of intra-group comparison showed that there was no significant difference in the scores of the intervention group before and after the intervention, and the difference was not statistically significant (*P*=0.32). After the experiment, the vital capacity scores of boys and girls in APP intervention group and control group were improved, with statistical significance (*P* < 0.05). The conclusion shows that running APP can improve students' speed level, cultivate students' endurance level, and improve students' physical health.

## 1. Introduction

Physical health education is especially important for college students because they are in the middle and late stages of growth and development. Universities are beginning to pay attention to students' physical quality as a result of the Ministry of Education's promotion of quality education, the definition of talents, and the demands of employers. It is not even close to that of senior high school students in many indicators, which is concerning. Mobile phone intelligence and running APP software are widely used in college students' extracurricular physical exercises in this era of rapid Internet development.

The unique function of running APP attracts the attention of college students, so that they can cultivate their correct exercise habits [1]. Jiang et al.'s survey of college students shows that 89.3% of boys like physical exercise, 68.1% of girls like physical exercise, and 10.7% of boys feel below average; girls accounted for 30.6%, which shows that girls' interest in physical exercise is slightly worse than that of boys [2]. Liu et al. pointed out that most students hold a good attitude toward exercise, but according to grades, the scores of exercise attitude vary from grade to grade, and the scores of lower grades are generally better than those of higher grades [3]. Kim et al. found through the experimental intervention of aerobics that aerobics has a positive effect on improving the oxidation strength of body fat. At the same time, the intervention program can also improve the body shape of female college students, effectively reduce the detection rate of female obesity, and help to improve the cardiopulmonary function [4]. O'Brien et al. found that women are twice as likely to give up engaging in sports activities and sedentary lifestyle as others [5]. Son et al. found that the physical health test level of students showed a downward trend. In terms of body shape, the number of obese boys decreased and the number of low-weight women increased. Physical function: The number of male and female students who passed the vital capacity test decreased [6].

The article "Analysis of Improving Effect of Running APP on College Students' Physique by Using Student Data Mining Technology" was retracted in 2023. Reasons: suspected computer-generated content; unreliable results or conclusions; lack of ethics approval or compliance; missing or withdrawn patient consent.

To summarize, many scholars at home and abroad have conducted common research on attitudes toward physical exercise and have unique perspectives, but there are few studies on the changes in college students' physique and exercise attitudes before and after using the exercise APP. Data mining (DM) [7] is a new technology that combines several disciplines and serves as a decision-making aid. This study looks at the impact of combining running apps with traditional physical education classes on college students' physical health, and as a result, it uncovers a new approach to college physical education that has a positive impact on promoting college students' physical exercise behavior, increasing their awareness of the benefits of exercise, and developing their physical exercise habits.

Innovation of research:

1. This study starts with the impact of running apps on college students' physical health and studies the benefits of sports apps on college students' physical health, which can provide theoretical and practical basis for college physical education workers to carry out physical education reform.
2. This paper attempts to apply DM technology to the analysis of college students' physique improvement effect, in order to dig out useful knowledge hidden in the data of college students' physique improvement effect through the application of DM technology and use these valuable knowledge to accurately predict college students' physique health status, so as to provide scientific basis for the planning and decision-making of physique health education.

The article "Analysis of Improving Effect of Running APP on College Students' Physique by Using Student Data Mining Technology" was retracted in 2023. Reasons: suspected computer-generated content; unreliable results or conclusions; lack of ethics approval or compliance; missing or withdrawn patient consent.

## 2. Related Work

### 2.1. Review of Sports APP-Like Research

The application of running APP has attracted the attention and recognition of sports lovers and scholars, highlighting the trend of intelligent development. The use of running app has gradually developed into a fashion and trend in the current society. Üner et al. found that the use of sports APP can promote college students' extracurricular physical exercise, and they can share their sports achievements through the APP to get a sense of accomplishment, thus prompting students to participate in physical exercise every day and develop good sports habits [8]. Eljko et al. found that sports APP can improve students' interest in exercise and stimulate students' persistence in exercise, and many advantages can promote exercisers to develop good habits in physical exercise [9]. Lv et al. conducted a survey on college students using sports apps and found that the reward mechanism, sense of achievement, and social function of sports apps can stimulate students' potential sports needs, and at the same time, they can also play a positive role in improving students' interest in physical exercise and enhancing their awareness and behavior of physical exercise [10].

Dol et al. found through research that the use of after-school running APP has a significant impact on students' body shape. This activity can help students lose weight and keep a normal body shape [11]. Wang et al. conducted a two-semester experiment on 286 students who used the running APP in Normal University. Through the comparison of physical fitness test results, they found that the students' height did not change much, and insisting on physical exercise would improve their vital capacity to a certain extent [12]. Yang et al. used the experimental control method to investigate the influence of mobile APP fitness software on college students' physical fitness level. The students in APP intervention group took online exercise intervention for 3 months, while the students in control group kept routine life. After the intervention, the vital capacity level of APP intervention group students was significantly higher than that of the control group, and the respiratory system function was also better than that of the control group students [13]. Tao found through comparing the students' physical health test results before and after using: all the data of students' physical fitness indexes have changed greatly, and the increase rate is obviously greater than the decrease rate, which shows that running APP can obviously promote the improvement of students' physical fitness [14].

The article "Analysis of Improving Effect of Running APP on College Students' Physique by Using Student Data Mining Technology" was retracted in 2023. Reasons: suspected computer-generated content; unreliable results or conclusions; lack of ethics approval or compliance; missing or withdrawn patient consent.

### 2.2. DM Research

The students' physical health detection system based on DM overcomes many limitations of traditional manual detection by using modern computer technology, transfers the traditional detection form to the computer, adopts information technology, and uses the computer to complete the detection efficiently and accurately.

Carey et al. applied AR (association rule) to DM them, taking individual indexes of physical fitness test as input and overall physical fitness score as output, and found that the indexes that have great influence on college girls' physical fitness are speed, flexibility, and vital capacity [15]; Xue et al. used an array-based Apriori algorithm to mine and analyze the physical fitness test items of college students, found out the correlation of each test item, and judged the rationality of each test item setting [16]. Liu et al. used the Apriori algorithm of AR and set the thresholds of support, confidence, and promotion to screen out the strong AR of boys' and girls' data, respectively, and got the test index that “the total score is equal to passing” [17]. Chen et al. investigated college students by questionnaire and physical fitness test, built a database, and built an ARDM model with physical exercise behavior stage as the output and physical fitness index as the input. The results show that the physical fitness of male students in the expected stage is mainly manifested as low cardiopulmonary function, moderate reaction time and excellent hands back hook, and low cardiopulmonary function, strength quality, and reaction time difference in preparation stage [18].

Aggarwal et al. took college students' physique test data as an example, introduced the concept of trend selection, and applied DT (decision tree) algorithm to the analysis of physique test data. This research combined the advanced DM algorithm [19], improved the accuracy, and achieved the purpose of monitoring students' physique to a certain extent. Zhang et al. used DM technology to mine a large amount of accumulated historical data, trying to find out the factors that affect school sports research and teaching and training, and using the relationship between these factors to discover sports talents. For the data analysis of physical health test, Yuan and Chen et al. studied the application of ARDM technology in system test analysis [20].

## 3. Methodology

### 3.1. Introduction to DM Technology

DM is the process of extracting implicit, unknown but potentially useful information and knowledge from a large number of incomplete, noisy, chaotic, and random data [9]. The knowledge that DM can extract can generally be divided into general knowledge, characteristic knowledge, difference knowledge, association knowledge, deviation knowledge, prediction knowledge, etc. AR is a rule that states that the values of two or more data items in a data set have a certain relationship or interaction. Changes in the value of one or more data items, for example, will cause changes in another or more data elements. Clustering [21, 22] is the process of summarizing and grouping data objects into various classes or groups based on the principle of maximizing class similarity while minimizing class similarity. Objects belonging to the same class are very similar, but objects belonging to different classes are very different. Sorting is one of the most important tasks in DM. Its main process is as follows: firstly, the training set of classification is selected from the database, the classification model is established on the basis of the training set by using the classification technology, and then the data items in the database are assigned to a certain category in a class. It can be applied to customer classification, customer characteristics and attribute analysis, customer purchase trend prediction, etc. Generally, data classification can be summarized into two steps: building a model and classifying using the model, as shown in Figure 1.

The article "Analysis of Improving Effect of Running APP on College Students' Physique by Using Student Data Mining Technology" was retracted in 2023. Reasons: suspected computer-generated content; unreliable results or conclusions; lack of ethics approval or compliance; missing or withdrawn patient consent.

Each tuple in the default data set has a class label; that is, it belongs to a default class. The model is built by parsing the attribute description of the tuple from the database. Usually, the first step of learning is used to build a model in the form of DT, formula, or rule. This model can be used to classify other samples and provide a deeper understanding of the database. Using each test sample in the test data set, the predicted categories learned by the classification model are compared with the known category labels. If it is the same, the sorting is successful; if they are different, the classification is unsuccessful.

### 3.2. Student DM Model Construction

#### 3.2.1. AR Modeling

Physical inactivity poses a number of health risks. The quantification of physical activity, regardless of the method used, will have no significant impact. However, a thorough understanding of the factors that contribute to a lack of physical activity can lead to targeted solutions. Furthermore, perceived barriers may be a result of external factors such as a lack of support from friends and family, safety concerns, limited transportation options, or a lack of time due to other obligations. Seasonal effects are another example of environmental barriers. Reluctance to participate in sports or sports activities because of the weather is one example [12]. In China, most scholars assess students' physical health based on three factors: body shape, physical function, and physical quality. On the one hand, the Ministry of Education's monitoring results of students' physical health have provided a comprehensive evaluation and analysis of the physical health of college students, the health development trend of students. However, urban students' average height, weight, and bust are higher than rural students', and boys are taller than girls. The rates of underweight and malnutrition have decreased, and students' nutritional status has improved over time. The added value of height, weight, and bust is higher for rural students than for urban students.

The article "Analysis of Improving Effect of Running APP on College Students' Physique by Using Student Data Mining Technology" was retracted in 2023. Reasons: suspected computer-generated content; unreliable results or conclusions; lack of ethics approval or compliance; missing or withdrawn patient consent.

ARDM input field type is usually required to be numeric. The ARDM aims to find out the physical health status of college students in different stages of sports behavior, so the output field is “physical exercise behavior” and the input field is “body mass index,” which constitutes the mapping relationship between “physical exercise,” “behavior,” and “health index.” This paper establishes a model of “association mining law between physical exercise behavior and individual indicators,” discusses the influence of physical exercise behavior on physical fitness, and provides decision support for the physical health of college students with different physical exercise behaviors. AR mining refers to finding the correlation between certain information from massive data. In short, it is to find out which transactions always happen at the same time or have a high probability of happening at the same time. The support degree can be expressed as

(1) $$\begin{array}{c} \text{support}\left(X\;\Rightarrow \;Y\right). \end{array}$$

Namely, support(*X* ⇒ *Y*)=support *X* ∪ *Y*=*P*(*X*, *Y*), which means the proportion of the number of transactions containing *X*, *Y* in the whole transaction set.

Assuming *I*_1_, *I*_2_ ⊆ *I*; *I*_1_∩*I*_2_=∅, then the credibility of AR can be expressed as

(2) $$\begin{array}{c} \text{Confidence}\left(I_{1}\;\Rightarrow \;I_{2}\right)=\frac{\text{support}\left(I_{1}\cup I_{2}\right)}{\text{support}\left(I_{1}\right)}. \end{array}$$

It refers to the ratio of the number of things containing *I*_1_, *I*_2_ to the number of things containing *I*_1_.

AR is an implicit formula shaped like *I*_1_ ⇒ *I*_2_, where *I*_1_, *I*_2_ is called the forerunner and successor of AR, respectively [21].

The confidence of AR is the number of transactions including both *X* and *Y* in the transaction set and the ratio of all transactions to those including *X*, which is Confidence(*X* ⇒ *Y*), and is expressed by the formula

(3) $$\begin{array}{c} \text{Confidence}\left(X\;\Rightarrow \;Y\right)=\frac{\text{support}\left(X\cup Y\right)}{\text{support}\left(X\right)}=P\left(Y\;|\;X\right). \end{array}$$

The main function of confidence is to describe the probability of *Y* when transaction *X* happens.

The article "Analysis of Improving Effect of Running APP on College Students' Physique by Using Student Data Mining Technology" was retracted in 2023. Reasons: suspected computer-generated content; unreliable results or conclusions; lack of ethics approval or compliance; missing or withdrawn patient consent.

In order to improve the mining efficiency, it is necessary to further simplify the data set, that is, to remove useless data according to the mining task and determine the data set for mining. Try not to use Chinese characters. Those Chinese attribute values can be replaced by English characters, numbers, or a combination of English characters and numbers. Apriori algorithm can be used to analyze the preprocessed data to find some hidden AR in the data. This rule infers the preprocessed transaction information to construct Bayesian DM model.

Suppose there is a rule condition *Q* and a rule conclusion *D*, where *D* represents an element in the peer relation set *θ*_*Q*_ of rule condition *Q* and *Y*_*j*_ represents an element in the peer relation set *θ*_*D*_ of rule conclusion *D*. A standardized function can be obtained, as shown in formula

(4) $$\begin{array}{c} S\left(D\;|\;Q\right)=1-\frac{H\left(D\;|\;Q\right)}{\log_{2}\left(n\right)}. \end{array}$$

The closer the value of *S*(*D* *|* *Q*) is to 1, the more similar the information contained in *D*, *Q* is, and the stronger the correlation between them. On the contrary, the closer the value of *S*(*D* *|* *Q*) is to 0, the more different the information contained in *D*, *Q* is.

Suppose there is one user, and its corresponding Bayesian DM model is shown in Figure 2.

From the recommendation results of the global recommendation model, select the only one added to the personal recommendation list, and the physical fitness test items in the associated list are sorted according to the probability value; that is, the higher the physical fitness test, the higher the chance of being selected.

#### 3.2.2. DT Structure

The essence of DT induction is to use a series of rules to classify the analyzed data. Most DT algorithms are greedy algorithms, starting with the training sample set and its related class labels, and constructing DT in a recursive top-down divide-and-conquer way [15]. Finally, the path from the root node at the top of the model to the leaf node at the bottom is a classification rule. C5.0 is a classical algorithm in DT model [21]. C5.0 DT growth process adopts the principle of maximum information gain rate to select nodes and split points. The weighted sum of the entropy of the split node minus the entropy of the split child node means that the impurity decreases; that is, the purity increases. The formula is

(5) $$\begin{array}{c} \text{Gain}=\text{Info}-{\text{Info}}_{A}. \end{array}$$

Infois the information entropy of *Y* variable, and Info_*A*_ is the information entropy of independent variable *A* dividing *Y* variable. The formula is

(6) $$\begin{array}{c} {\text{Info}}_{A}=-\sum_{j=1}^{v}p_{j}\text{Info}\left(A_{j}\right),p_{j}=\frac{N_{j}}{N}. \end{array}$$

Because the information gain selection is biased toward attributes with more values (the more the values of parameters, the higher the purity of sub-nodes after segmentation). C5.0 uses the method of information gain rate to balance discrete variables with relatively few levels [17].

The article "Analysis of Improving Effect of Running APP on College Students' Physique by Using Student Data Mining Technology" was retracted in 2023. Reasons: suspected computer-generated content; unreliable results or conclusions; lack of ethics approval or compliance; missing or withdrawn patient consent.

The expected information required to classify tuples in *R* according to attribute *A* is defined as

(7) $$\begin{array}{c} {\text{Info}}_{A}\left(R\right)=-\sum_{i=1}^{m}\frac{\left|C_{i}\right|}{R}\cdot \text{Info}\left(C_{i}\right). \end{array}$$

The information gain of *A* to *R* is defined as

(8) $$\begin{array}{c} {\text{Gain}}_{A}=\text{Info}\left(R\right)-{\text{Info}}_{A}\left(R\right). \end{array}$$

Attribute selection metric is the criterion for selecting classifications. Which attribute is used for each classification during DT construction? Its purpose and judgment criterion is to divide a given training tuple data set into the “best” subclass. Ideally, all tuples falling into a given partition belong to the same class.

In this way, many branches are established based on the anomalies in the sample set, resulting in over-fitting of the generated DT to the training samples. In order to solve the above data over-fitting problem and obtain more general classification rules, it is necessary to prune the generated DT model directly. The specific implementation of pruning is to cut off each branch according to a certain pruning algorithm and then replace it with leaves. After pruning, DT becomes smaller and less complicated, so the generated rules are easier to understand [19]. Among several pruning algorithms, this paper selects PEP (pessimistic error pruning) algorithm to prune students' DM models. *T* represents the original tree; *T*_*t*_ represents the subtree at the node with node *t* as the root; *e*(*t*) represents the number of misclassified instances at node *t*; *n*(*t*) represents the number of all instances covered at node *t*.

The classification error rate at node *t* is

(9) $$\begin{array}{c} r\left(t\right)=\frac{e\left(t\right)}{n\left(t\right)}. \end{array}$$

PEP algorithm corrects it to

(10) $$\begin{array}{c} r^{\prime }\left(t\right)=\frac{e\left(t\right)+1/2}{n\left(t\right)}. \end{array}$$

The standard error *SE*[*e*′(*T*_*t*_)] is defined as

(11) $$\begin{array}{c} SE\left[e^{\prime }\left(T_{t}\right)\right]=\sqrt{\frac{e^{\prime }\left(T_{t}\right)\left[n\left(t\right)-e^{\prime }\left(T_{t}\right)\right]}{n\left(t\right)}}. \end{array}$$

PEP algorithm is faster and more efficient than other algorithms because each subtree is accessed at most once during pruning, and it is recognized as one of the most accurate pruning algorithms. PEP algorithm is used to identify the class labels of leaf nodes and the classes to which most samples belong in the downward pruning subtree. Finally, the DM student model based on PEP pruning is constructed as shown in Figure 3.

The article "Analysis of Improving Effect of Running APP on College Students' Physique by Using Student Data Mining Technology" was retracted in 2023. Reasons: suspected computer-generated content; unreliable results or conclusions; lack of ethics approval or compliance; missing or withdrawn patient consent.

Obviously, the scale of the pruned DT model is smaller than that of the directly generated DT model, which can directly improve the readability of the DT model and the classification speed of new data.

## 4. Experiment and Results

### 4.1. Knowledge Discovery and Decision Support of Physical Health of Male and Female Students

Taking the stage of physical exercise behavior as the output, the maximum number of rules is 6, and 18 pieces of knowledge are found. After screening, a total of 7 pieces of knowledge that are important for decision-making were found. The AR knowledge found by boys is shown in Table 1.

In the action stage, the boys found three meaningful pieces of knowledge through AR. No. 7' knowledge was “excellent” when he answered. Knowledge support is 7.874%, and confidence is 56.387%. Compared with No. 6 knowledge, it shows that physical exercise can positively and effectively improve boys' knowledge and flexibility of nervous system. Therefore, for the boys who actively take part in physical exercise, we should guide their scientific exercise pertinence, strengthen the exercise prescription, focus on the development of cardiopulmonary function and strength exercise, and cultivate their hard-working spirit psychologically.

The discovery of AR knowledge of girls is shown in Table 2.

There are three knowledge findings that can be used to support girls' decision-making in the action stage. The physical characteristics of girls at this stage are low strength, moderate reaction time, and good flexibility. Because from the age point of view, all indicators of girls should be in the “peak” period, but this is not the case, which shows that girls at this stage have already learned the relevant knowledge of physical health and look forward to improving their physical fitness, so that they can get healthy through physical exercise.

### 4.2. Comparative Results of College Students' Physical Fitness

The comparison results of 1000 m grades of boys in the APP intervention group and the control group are shown in Figure 4.

The results showed that after 10 weeks of intervention, there was a significant difference between the 1000 m scores of the intervention group and the control group, and the scores of the intervention group were better than those of the control group, with statistical significance (*P*=0.007). The results of intra-group comparison showed that there was no significant difference in the score of 1000 m between the intervention group and the preintervention group (*P*=0.516). However, the 1000 m performance of the control group was significantly lower than that before the intervention, and the difference was statistically significant (*P*=0.001). See Table 3 for details.

The article "Analysis of Improving Effect of Running APP on College Students' Physique by Using Student Data Mining Technology" was retracted in 2023. Reasons: suspected computer-generated content; unreliable results or conclusions; lack of ethics approval or compliance; missing or withdrawn patient consent.

The comparison results of 800 m grade of girls in APP intervention group and control group are shown in Figure 5 and Table 4.

The results showed that after 10 weeks of intervention, the 800 m scores of girls in the intervention group were significantly different from those in the control group. The 800 m scores of girls in the intervention group were better than those in the control group, and the difference was statistically significant (*P*=0.03). The results of intra-group comparison showed that there was no significant difference in scores before and after intervention in the intervention group (*P*=0.32), but there was significant difference in scores after intervention in the control group. The difference was statistically significant (*P*=0.001).

### 4.3. Research Result of College Students' Physical Function Index

The comparison results of physical function indexes between APP intervention group and control group after the experiment are shown in Table 5.

Through the independent sample *T*-test of physical function index data of APP intervention group and control group after experiment, it can be seen from Table 4 that the vital capacity scores of boys and girls in APP intervention group and those in control group improved after experiment, with statistical significance, *P* < 0.05. It shows that a 12-week exercise intervention in the form of running with the help of running APP software has a positive effect on improving students' vital capacity performance.

### 4.4. Comparison of Students' Exercise Attitudes after Using APP

Most college students are aware of the importance of physical exercise to their own health, but few people actually put it into practice. It can be seen that college students' sports cognition level is not in harmony with their own practice level. With the profound understanding of college students' sports values, many college students begin to attach importance to physical exercise and are willing to devote their time to sports.  Figure 6 shows the distribution of college students' attitudes toward sports plans with and without running apps on campus.

The article "Analysis of Improving Effect of Running APP on College Students' Physique by Using Student Data Mining Technology" was retracted in 2023. Reasons: suspected computer-generated content; unreliable results or conclusions; lack of ethics approval or compliance; missing or withdrawn patient consent.

As can be seen from Figure 6, students who use the running APP do not want the running APP to make a scientific exercise plan, accounting for 38%, while 111 students who do not use the running APP do not want to use the running APP, accounting for 62%. The survey results show that most students hope to have a scientific exercise plan to guide them to exercise. In order to explore whether there are differences in exercise attitudes among boys after using APP, this study conducted independent sample *T*-test on the scores of exercise attitudes of school boys, and the statistical results are shown in Figure 7.

As can be seen from Figure 7, the average score of boys' exercise attitude using APP is 260.39 points, and that of boys' exercise attitude not using APP is 233.19 points. There is a very significant difference between them (*P* < 0.01). It shows that the exercise attitude of boys using APP is obviously better than that of boys not using APP. In order to explore whether there are differences in girls' exercise attitudes after using APP, this study conducted independent sample *T*-test on school girls' exercise attitude scores, and the statistical results are shown in Figure 8.

As can be seen from Figure 8, the average score of girls' exercise attitude using APP is 235.49 points, and that of girls' exercise attitude not using APP is 231.64 points. There is a significant difference between them (*P* < 0.05). It shows that the exercise attitude of girls using APP is obviously better than that of girls not using APP. Through comparative analysis, the sports attitude of the students who use APP is better than that of the students who do not use APP, and there is no significant difference in the four dimensions of “goal attitude,” “behavior attitude,” “cognition,” and “emotional experience.” There are very significant differences in other dimensions. Girls who use it have a better attitude toward sports than those who do not. It is mainly manifested in “behavior control,” “habitual behavior,” and “subjective standard.” Girls who use APP are more automatic in physical exercise, have strong self-control ability in physical exercise, and are more willing to make greater efforts for physical exercise.

To sum up, after 10 weeks of APP running intervention, the aerobic endurance of boys and girls has not improved significantly, which may be related to the normal performance of APP running evaluation standard. In addition, it may be related to the short intervention time. It shows that running APP software for 10 weeks can effectively improve students' breathing depth, the functional state of respiratory system, and their vital capacity. At the same time, students can participate in competitions with friends and classmates through running, communication, and other running APP functions, thus satisfying students' enthusiasm for participating in sports, allowing them to participate in physical exercise activities, be independent, and experience physical exercise activities better.

The article "Analysis of Improving Effect of Running APP on College Students' Physique by Using Student Data Mining Technology" was retracted in 2023. Reasons: suspected computer-generated content; unreliable results or conclusions; lack of ethics approval or compliance; missing or withdrawn patient consent.

## 5. Conclusions

This paper draws the following conclusions based on the analysis of the effect of a running APP based on students' DM on college students' physical fitness: (1) the APP intervention group's changes in two physical fitness indexes, 800 m and 1000 m, are clearly better than before the exercise intervention, but there is no significant difference in the control group's physical fitness indexes. It demonstrates that using APP software improves the speed quality of college students. (2) The vital capacity scores of boys and girls in the APP intervention group and the control group improved after the experiment, with statistical significance (P0.05). It demonstrates that a 12-week exercise intervention in the form of running using running APP software can help students improve their vital capacity. (3) The APP intervention has a clear effect on improving the vital capacity of male students. It effectively slowed the decline in female students' vital capacity to some extent. College students' attitudes toward exercise have clearly changed after using the running APP. Whether it is boys or girls, the exercise attitude of those who use the running APP is clearly superior to those who do not.

## Figures and Tables

**Figure 1:** Classification steps.

**Figure 2:** Bayesian model.

**Figure 3:** Student DM model based on PEP pruning.

**Figure 4:** Comparative result.

**Figure 5:** Comparison of 800 m grade between intervention group and control group.

**Figure 6:** Attitudes of college students who use running APP and those who do not use running app toward sports plan.

**Figure 7:** Comparison of boys' exercise attitudes after using APP.

**Figure 8:** Comparison of girls' exercise attitudes after using APP.

**Table 1:** AR knowledge discovery of boys.

Serial number	AR	Support (%)	Confidence (%)
1	Left back hook ⟶ excellent, body fat rate ⟶ normal	9.327	50.221
2	Left back hook ⟶ excellent, reaction time ⟶ medium	9.704	50.014
3	Grip strength ⟶ difference	9.161	51.006
4	Reaction time ⟶ difference	8.445	66.367
5	Reaction time ⟶ excellence	8.346	60.221
6	Reaction time ⟶ good reaction	8.407	90.168
7	Reaction time ⟶ good, grip strength ⟶ poor	7.874	56.387

**Table 2:** Girls' AR knowledge discovery.

Serial number	AR	Support (%)	Confidence (%)
1	Right back hook ⟶ excellent, grip strength ⟶ poor	10.367	66.538
2	Reaction time ⟶ medium, right back hook ⟶ excellent	12.126	74.152
3	Body fat rate ⟶ overweight	13.015	66.628
4	Right back hook ⟶ excellent	10.069	63.012
5	Reaction time ⟶ medium, right back hook ⟶ excellent	10.015	70.014
6	Grip strength ⟶ poor, body fat rate ⟶ overweight	11.225	68.963
7	Grip strength ⟶ difference	12.638	66.248

The article "Analysis of Improving Effect of Running APP on College Students' Physique by Using Student Data Mining Technology" was retracted in 2023. Reasons: suspected computer-generated content; unreliable results or conclusions; lack of ethics approval or compliance; missing or withdrawn patient consent.

**Table 3:** Comparison of boys' 1000 m running results between intervention group and control group (*N* = 160, unit: s).

	Intervention group	Control group
Before intervention	244.53 ± 22.53	240.14 ± 20.69
After intervention	249.13 ± 35.62	266.38 ± 56.79

**Table 4:** Comparison of girls' 1000 m running results between intervention group and control group (*N* = 160, unit: s).

	Intervention group	Control group
Before intervention	246.41 ± 44.12	245.39 ± 42.01
After intervention	253.66 ± 26.41	266.38 ± 23.68

**Table 5:** Comparison results of vital capacity experiment (*N* = 160).

Gender	Before intervention	After intervention	T	*P*
Man	3887.96 ± 897.21	4233.87 ± 566.85	−2.46	0.03^*∗*^
Woman	2863.28 ± 412.33	2986.17 ± 378.56	−2.33	0.02^*∗*^

*Note.* “^*∗*^” means that *P* < 0.05 is a significant difference.

## Data Availability

The data used to support the findings of this study are available from the corresponding author upon request.
